# Clinical Data-CT Radiomics-Based Model for Predicting Prognosis of Patients with Gastrointestinal Pancreatic Neuroendocrine Neoplasms (GP-NENs)

**DOI:** 10.1155/2022/4186305

**Published:** 2022-08-05

**Authors:** Peng An, Junyan Zhang, Mingqun Li, Peng Duan, Zhibing He, Zhongq Wang, Guoyan Feng, Hongyan Guo, Xiumei Li, Ping Qin

**Affiliations:** ^1^Department of Radiology, Xiangyang No.1 People's Hospital, Hubei University of Medicine, Xiangyang 441000, China; ^2^Department of Pharmacy and Laboratory, Xiangyang No.1 People's Hospital, Hubei University of Medicine, Xiangyang 441000, China; ^3^Department of Internal Medicine, Xiangyang No.1 People's Hospital, Hubei University of Medicine, Xiangyang 441000, China; ^4^Department of Oncology/Obstetrics and Gynecology, Xiangyang No.1 People's Hospital, Hubei University of Medicine, Xiangyang 441000, China; ^5^Department of Radiology, The Affiliated Hospital of Nanjing University of Chinese Medicine, Jiangsu Province Hospital of Chinese Medicine, The First Clinical Medical College, 155 Hanzhong Road Nanjing, 210029 Jiangsu Province, China

## Abstract

**Purpose:**

Based on computerized tomography (CT) radiomics and clinical data, a model was established to predict the prognosis of patients with gastrointestinal pancreatic neuroendocrine neoplasms (GP-NENs).

**Methods:**

In the data collection, the clinical imaging and survival follow-up data of 225 GP-NENs patients admitted to Xiangyang No.1 People's Hospital and Jiangsu Province Hospital of Chinese Medicine from August 2015 to February 2021 were collected. According to the follow-up results, they were divided into the nonrecurrent group (*n* = 108) and the recurrent group (*n* = 117), based on which a training set and a test set were established at a ratio of 7/3. In the training set, a variety of models were established with significant clinical and imaging data (*P* < 0.05) to predict the prognosis of GP-NENs patients, and then these models were verified in the test set.

**Results:**

Our newly developed combined prediction model had high predictive efficacy. Univariate analysis showed that Radscore 1/2/3, age, Ki-67 index, tumor pathological type, tumor primary site, and TNM stage were risk factors for the prognosis of GP-NENs patients (all *P* < 0.05). The area under the receiver operating characteristic (ROC) curves (AUC) of the combined model was significantly higher [AUC:0.824, 95% CI 0.0342 (0.751-0.883)] than that of the clinical data model [AUC:0.786, 95% CI 0.0384(0.709-0.851)] and the radiomics model [AUC:0.712, 95% CI 0.0426(0.631-0.785)]. The decision curve also confirmed that the combined model had a higher clinical net benefit. The same results were achieved in the test set.

**Conclusion:**

The prognosis of patients with GP-NENs is generally poor. The combined model based on clinical data and CT radiomics can help to early predict the prognosis of patients with GP-NENs, and then necessary interventions could be provided to improve the survival rate and quality of life of patients.

## 1. Introduction

Gastrointestinal pancreatic neuroendocrine neoplasms (GP-NENs) are a rare malignancy derived from gastrointestinal neuroendocrine cells [1, 2]. The incidence of GP-NENs has been rising in recent years due to factors such as poor dietary habits, heredity, excessive stress, and environmental pollution in China [3, 4]. According to the degree of differentiation, the World Health Organization (WHO) classifies GP-NENs into two categories, well-differentiated gastrointestinal pancreatic neuroendocrine tumor (GP-NET) and poorly differentiated gastrointestinal pancreatic neuroendocrine carcinoma (GP-NEC). According to the 8th edition of American Joint Committee on Cancer (AJCC) staging system for GP-NENs, GP-NET and GP-NEC are very different in biological characteristics, tumor malignancy, and prognosis [5, 6]. It is reported that the pathological type of tumor and TNM stage are risk factors for prognosis; but these factors are more one-sided and will be interfered by pathological section technology and human factors. However, at present, the prognosis of some special cases cannot be identified simply by the pathological assessment standard of AJCC. Our team often found false-negative cases with poor prognosis. Therefore, the effect of the previous prediction model is poor. Moreover, there were few studies on this issue reported in PubMed for the last 40 years, and most studies focused on pathological classification and clinical treatment (Figure 1). As a result, there is still a lack of a comprehensive prognostic prediction system for GP-NENs [7, 8]. Therefore, this study aimed to establish a predictive model for the prognosis of GP-NENs based on clinical imaging data, to provide a new method for individualized clinical decision-making for GP-NEN patients and to increase the survival rate of patients (Figure 2).

## 2. Materials and Methods

### 2.1. Case Data

The clinical imaging and survival follow-up data of 244 patients who were pathologically diagnosed with GP-NENs in Xiangyang No.1 People's Hospital and Jiangsu Province Hospital of Chinese Medicine from August 2015 to February 2021 were collected, including gender, age, tumor pathological type, tumor primary site, TNM stage, Ki-67 index, and radiomics parameters for three contrast-enhanced computerized tomography (CT) phases. The inclusion criteria were with complete GP-NENs clinicopathological and imaging data and with complete follow-up data. The exclusion criteria were patients with GP-NENs metastases with primary cancer in other organs, or combined with other tumors, or combined with major organ dysfunction [9] (Figure 3).

### 2.2. CT Scanning and Radiomics Methods

The plain and contrast-enhanced abdomen CT scans were performed using the Siemens SOMATOM Definition Edge 64-slice/Sensation 64-slice CT. The patient was asked to drink 500 ml of water on an empty stomach within 0.5 h before the scan to fill the stomach cavity, and the patient was in a supine position during scanning. CT scanning parameters were as follows: tube voltage 80 kVp/140 kVp fast switching, automatic milliamp second, rotation speed 0.6 s/r, fixed tube current 600 mA, pitch 0.983, collimator width 0.625 mm, and reconstruction slice thickness and interval 1.25 mm. The contrast agent was ioversol (320 mgI/ml), at a flow rate of 3~4 ml/s and with a dose of 1.0 ml/kg, and was bolus injected through an anterior cubital vein using a high-pressure syringe. The arterial phase scan was automatically initiated. Followed with a delay of 25~30 s, the venous phase was obtained. Followed with another delay of 50~60 s, the delay phase was obtained [10, 11].

### 2.3. Radiomics Analysis Process

In this study, 3D slicer (version 4.11.20210226, https://www.slicer.org/) image segmentation software was used to delineate the region of interest (ROI) of GP-NENs masses, including plain scan, arterial phase, and venous phase CT data, and followed by texture analysis and data extraction. After determining the candidate texture data such as firstorder, glcm, and ngtdm, R (version 4.1.3) was then used to perform cross-validation and Lasso coefficients regression on the above texture data to extract valid texture data and generate radiomic score (Radscore) values [12, 13].

### 2.4. Statistical Methods

All data were first analyzed using SPSS 22.0. The measurement data subjected to normal distribution were expressed as mean ± standard deviation(*x* ± *s*), and the independent samples *t*-test was used to conduct between-group comparison. The *χ*2 test or Fisher's exact test was used to compare the count data between groups. The rank-sum test was used to analyze nonnormally distributed data. Then, multiple regression analysis was performed to calculate the odds ratio (OR) and 95% confidence interval (95% CI), with *P* < 0.05 indicating statistically significant differences. R was used to establish the training set and test set at a ratio of 7/3. In the training set, the clinical data model, the radiomics model, and the combined model were established based on the statistically significant clinical data, CT radiomics data, and both data using logistic regression (*P* < 0.05), respectively. Then the receiver operating characteristic (ROC) curves of the three models were made, and the areas under the ROC curves (AUCs) were calculated to evaluate the performance of the models to predict the prognosis of GP-NENs. Furthermore, the predictive performance of the models was evaluated on the test set. Decision curve analysis (DCA) was performed on the training and test sets to determine their clinical usefulness by quantifying the net gain in the model at various threshold probabilities. The other statistical analyses were performed using R (https://www.r-project.org/) [14, 15].

## 3. Results

### 3.1. Analysis of Clinical Data

There were statistically significant differences in age, tumor pathological type, primary tumor site, Ki-67 index, TNM stage, lymph node metastasis, and distant metastasis between the two groups (all *P* < 0.05), while other factors like gender was not related to the prognosis of patients with GP-NENs (all *P* > 0.05) (Table 1).

Univariate regression analysis showed that age, tumor pathological type, primary tumor site, Ki-67 index, TNM stage, lymph node metastasis, and distant metastasis were risk factors for GP-NENs' poor prognosis. However, multivariate regression analysis showed that tumor pathological type, primary tumor site, Ki-67 index, TNM stage, and lymph node metastasis were independent risk factors for GP-NENs' poor prognosis.

### 3.2. Radiomics Results

Our team extracted a total of 2,622 sets of texture data from the ROIs of the GP-NENs mass delineated by 3D slicer software and then obtained a total of 55 sets of texture parameters based on the Lasso regression in R and eventually generated Radscore 1 (plain CT scan), Radscore 2 (CT-enhanced arterial phase), and Radscore 3 (CT-enhanced venous phase). In the subsequent analysis, Radscore 1/2/3 were shown to be significantly different between groups (*P* < 0.05) (Figure 4 and Table 2).

(1) $$\begin{array}{c} \text{Radscore }1=-0.676*\text{MeanAbsoluteDeviation}...329+0.239*\text{wavelet}‐\text{LLLglcmClusterShade}+-0.296*\text{DifferenceVariance}...104+0.38*\text{InterquartileRange}...326+-0.11*\text{Uniformity}...33+..\cdots +0.543*\text{wavelet}‐\text{HLHfirstorderMedian}+-0.243*\text{Idn}...413+-0.977*\text{MeanAbsoluteDeviation}...512+-0.137*\text{SmallDependenceHighGrayLevelEmphasis}...498+0.175*\text{Strength}\cdots 443+0.29*\text{SurfaceArea}+-0.063*\text{wavelet}‐\text{HHHfirstorderMean}+0.132,\\ \text{Radscore }2=\;-3.823*\text{MinorAxisLength}+-0.604*\text{MeanAbsoluteDeviation}...329+0.041*\text{Idn}...47+-0.886*\text{MeanAbsoluteDeviation}...512+-0.745*\text{wavelet}‐\text{HLLglszmSmallAreaEmphasis}+0.402*\text{SurfaceArea}+..\cdots +-0.126*\text{Idn}...413+-0.642*\text{GrayLevelVariance}...64+-0.445*\text{DependenceVariance}...428+-0.145*\text{wavelet}‐\text{HHHfirstorderMean}+-0.064*\text{SmallDependenceHighGrayLevelEmphasis}...498+-0.38*\text{Busyness}...134+0.66,\\ \text{Radscore }3=\;-2.949*\text{MinorAxisLength}+-0.924*\text{wavelet}‐\text{HLLglszmSizeZoneNonUniformityNormalized}+0.037*\text{wavelet}‐\text{LLLglcmClusterShade}+-0.518*\text{MeanAbsoluteDeviation}...329+0.244*\text{wavelet}‐\text{HLHfirstorderMedian}+..\cdots +-0.211*\text{Idn}...413+-0.097*\text{MeanAbsoluteDeviation}...146+-1.626*\text{MeanAbsoluteDeviation}...512+-0.449*\text{GrayLevelVariance}...64+0.43. \end{array}$$

Univariate regression analysis showed that Radscore 1, Radscore 2, and Radscore 3 were risk factors for GP-NENs' poor prognosis. However, multivariate regression analysis showed that Radscore 1 and Radscore 3 were independent risk factors for GP-NENs' poor prognosis.

### 3.3. Establishment and Verification of Various Prediction Models

Risk factors such as Ki-67 index, age, TNM stage, and Radscore 1/2/3 were included to construct the clinical data model, radiomics model, and combined model. As analyzed by MedCalc (version 20.0.22), the combined model demonstrated the best predictive performance [AUC:0.824, 95% CI 0.0342(0.751-0.883)], significantly higher than the clinical data model [AUC:0.786, 95% CI 0.0384(0.709-0.851)] and the radiomics model [AUC:0.712, 95% CI 0.0426(0.631-0.785)]. Furthermore, the subsequent DCA also confirmed that the net benefit of the combined model was significantly higher than other models. Moreover, the expected results were also verified in the test set, with the highest predictive efficiency by the combined model [AUC:0.885, 95% CI 0.0367(0.797-0.945)], significantly higher than the clinical data model [AUC:0.803, 95% CI 0.0445(0.715-0.892)] and the radiomics model [AUC:0.763, 95% CI 0.0531(0.657-0.851)] (Table 3 and Figures 5 and 6).

Multivariate regression analysis showed that Radscore 1/3, TNM stage, primary tumor site, and lymph node metastasis were independent risk factors for GP-NENs' poor prognosis after combining the above risk factors (Tables 1 and 2).

## 4. Discussion

GP-NENs usually originate from enterochromaffin-like (ECL) cells and clinically can manifest as benign, low-grade malignant, or even aggressive tumors. The etiology remains elusive. With the advancement of pathological techniques and neoadjuvant therapy, the diagnosis rate and incidence rate of GP-NENs are increasing. Due to the high recurrence rate of GP-NENs, how to improve the surgical resection rate and reduce the metastasis rate of GP-NENs has attracted more and more attention [16, 17]. As of now, the treatment indications, regimen selection, efficacy, and prognosis evaluation of neoadjuvant therapy in GP-NENs patients are still controversial, and its clinical application remains in the exploratory stage. Hence, the prognosis prediction before treatment is extremely important. Recently, Wang reported using a nomogram model based on the clinical data of GP-NENs to predict the prognosis of patients and achieved good prediction results [18, 19]. However, because of the individual differences in patients and differences in tumor growth patterns, this model could not find all the patients with GP-NENs recurrence [20, 21]. To solve this issue, the present study used the clinical imaging data of 225 patients for analysis, developed a more comprehensive predictive model, and achieved good clinical benefits.

In this study, it was revealed that age, pathological type, primary tumor site, Ki-67 index, TNM stage, and Radscores were related to the prognosis of GP-NENs. Among them, TNM stage and Radscores were the most sensitive parameters for the prognosis of GP-NENs. The details were as follows. (1) The older the patient, the poorer the body's tolerance, the lower the immunity, and the higher the risk of recurrence. (2) The higher the Ki-67 index, the higher the risk in prognosis. As reported, the Ki-67 index has been proven to be a marker of other various tumor recurrences; nevertheless, it works effectively for GP-NENs as well. (3) The TNM stage of the tumor is regarded as a classic tumor prognostic indicator. For patients with a high value in TMN stage and the primary tumor cannot be completely resected, bad prognosis was expected. For patients with complete resection of the primary tumor, the preoperative TMN stage was also an important indicator. (4) Distant metastasis and lymph node metastasis of GP-NENs were negatively correlated with the prognosis of patients. Local surgery or palliative treatment could not reverse the outcome in patients with metastases. (5) For pathological type of tumor, this study confirmed that GP-NEC patients had a worse prognosis than GP-NET. Poorly differentiated tumors have always been a potential factor for poor prognosis. (6) In the primary site of the tumor, we found that the prognosis of GP-NET originated from the pancreas was significantly worse than that originated from the gastrointestinal tract, probably related to the rapid progression of pancreatic tumors. Therefore, for patients with the above conditions, special attention should be paid to the possibility of GP-NENs progression [22, 23, 24].

Based on the above factors, we established a clinical data prediction model. However, subsequent data analysis showed inferior prediction accuracy of this model, with commonly false positive or false negative results. Therefore, we introduced the radiomics factor and obtained nice results. The concept of radiomics was first proposed by Lambin of the Department of Precision Medicine, Maastricht University, in the Netherlands in 2011. It refers to the high-throughput extraction of a large number of texture parameters describing tumor characteristics from CT/MRI (magnetic resonance imaging) and the establishment of a prediction model through machine learning to conduct deeper mining, prediction, and analysis on massive images features. As a noninvasive examination method, radiomics can extract a considerable amount of image features from medical images that cannot be seen by the naked eye, and it can be used to partially replace biopsy for prognosis evaluation and curative effect prediction [25, 26]. This study also extracted 2,622 sets of texture parameters based on the enhanced CT data of GP-NENs and obtained 3 sets of Radscores. The analysis results confirmed that the radiomics model (including Radscore 1/2/3) had better predictive performance. Presumably, this may be because that these parameters described the internal characteristics of the tumor. However, the radiomics model itself could not describe the clinical characteristics of patients. Therefore, we combined these two models to a combined model and obtained even better clinical benefit, which was significantly higher than the clinical data model and the radiomics model. Subsequent DCA also confirmed the combined model with a higher net benefit. And the same results were verified in the test set too, with the combined model significantly superior to the clinical data model and the radiomics model. In the end, the model was well received by the clinic.

## 5. Limitations

Nowadays, prediction models are widely applied in various clinical diseases, but their strict data differentiation requirements (*P* < 0.05) may make some potentially effective factors missed. Therefore, prediction models developed based on machine learning or artificial intelligence in the future will be more valuable. Secondly, we only used Lasso regression for the extraction of radiomics data, and this is not enough. Analysis adopting advanced algorithms will be included in the future [27, 28].

## 6. Conclusions

In conclusion, Radscore 1/3, TNM stage, primary tumor site, and lymph node metastasis were independent risk factors for prognosis of GP-NENs. It is feasible to establish a combined model based on clinical imaging data to predict the prognosis of patients with GP-NENs. In the future, we will conduct multicenter research to improve the predictive value of this model.

## Figures and Tables

**Figure 1:** From the content of references retrieval from 1982 to 2022, GP-NENs has always been a research hotspot, with more research on molecular mechanism, pathological classification, and clinical treatment but less on prediction of GP-NENs by multimodal radiomics models.

**Figure 2:** The technical flowchart of this study. Novelty of the work is a prediction model established using the enhanced CT radiomics combined with clinical data, which has not been reported before.

**Figure 3:** The simplified inclusion and exclusion criteria for patient enrollment in the present study.

**Figure 4:** Schematic diagram of radiomics texture feature extraction based on R Studio software (Lasso regression method), a total of 6 groups of available texture data are extracted; (a) the method of k-fold cross-verification by adjusting different parameters lambda (*λ*) filter out the characteristic parameter groups with the best performance. (b) The compression diagram of k-fold cross-validation method for screening characteristic parameters. The vertical black line is the best lambda value when the model performance is optimized. Notes: Radiomics scoring (Radscore) refers to the comprehensive expression and scoring of the extracted valuable radiomics texture parameters.

**Figure 5:** Delong nonparametric curves of the training set (a) and the test set (b). The area under the ROC curve of the combined model of the two groups is the largest;

**Figure 6:** The maximum net benefits of the combined model was confirmed in the two groups by DCA of training set (a) and test set (b) using R software.

**Table 1:** Logistic regression analysis results of clinical data model based on clinical characteristics for predicting the GP-NENs' prognosis, ∗*P* < 0.05.

Clinical data model	Univariate analysis		Multivariate analysis	
Factors	*P*	Hazard ratio	*P*	Hazard ratio
Gender	0.483	0.789 (0.408-1.529)		
History of hypertension	0.850	1.066 (0.551-2.060)		
Smoking history	0.268	0.684 (0.349-1.341)		
Drinking history	0.052	0.511 (0.259-1.007)		
Age	0.033∗	0.885 (0.791-0.990)		
Tumor pathological type	0.019∗	2.314 (1.150-4.657)	0.034∗	2.351 (1.067-5.181)
Primary tumor site	0.028∗	2.120 (1.083-4.149)	0.019∗	2.554(1.167-5.592)
Ki-67	0.015∗	1.040 (1.008-1.074)	0.022∗	1.043 (1.006-1.082)
TNM stage	0.012∗	2.386 (1.214-4.688)	0.044∗	2.215 (1.021-4.811)
Lymph node metastasis	0.030∗	1.118 (1.011-1.237)	0.019∗	1.163 (1.025-1.321)
Distant metastasis	0.026∗	1.164 (1.019-1.331)		
History of diabetes	0.861	1.061 (.549-2.049)		

**Table 2:** Logistic regression analysis results of radiomics model based on radiomics texture results for predicting the GP-NENs' prognosis, ∗*P* < 0.05.

Radiomics model	Univariate analysis		Multivariate analysis	
Factors	*P*	Hazard ratio	*P*	Hazard ratio
Radscore 1	0.004∗	1.006 (1.002-1.011)	0.007∗	1.006 (1.001-1.010)
Radscore 2	0.035∗	0.998 (0.996-1.000)		
Radscore 3	0.002∗	0.971 (0.952-0.989)	0.004∗	0.971 (0.952-0.991)

**Table 3:** Logistic regression analysis results of combined model based on mentioned valuable univariate regression analysis factors for predicting the GP-NENs' prognosis, ∗*P* < 0.05.

Combined model	Univariate analysis		Multivariate analysis	
Factors	*P*	Hazard ratio	*P*	Hazard ratio
Radscore 1	0.004∗	1.006 (1.002-1.011)	0.045∗	1.005 (1.001-1.011)
Radscore 2	0.035∗	0.998 (0.996-1.000)		
Radscore 3	0.002∗	0.971 (0.952-0.989)	0.021∗	0.974 (0.953-0.996)
Age	0.033∗	0.885 (0.791-0.990)		
Tumor pathological type	0.019∗	2.314 (1.150-4.657)		
Primary tumor site	0.028∗	2.120 (1.083-4.149)	0.035∗	2.481 (1.068-5.757)
Ki-67	0.015∗	1.040 (1.008-1.074)		
TNM stage	0.012∗	2.386 (1.214-4.688)	0.030∗	2.534 (1.093-5.872)
Lymph node metastasis	0.030∗	1.118 (1.011-1.237)	0.028∗	1.165 (1.017-1.334)
Distant metastasis	0.026∗	1.164 (1.019-1.331)		

## Data Availability

All data generated or analyzed during this study are included in this published article.
